This article has been retracted.

# Visual Identification of Mobile App GUI Elements for Automated Robotic Testing

**DOI:** 10.1155/2022/4471455

**Published:** 2022-04-23

**Authors:** Feng Xue, Junsheng Wu, Tao Zhang

**Affiliations:** ^1^School of Computer Science and Engineering, Northwestern Polytechnical University, Xi'an 710072, China; ^2^School of Software, Northwestern Polytechnical University, Xi'an 710072, China

## Abstract

Automated robotic testing is an emerging testing approach for mobile apps that can afford complete black-box testing. Compared with other automated testing approaches, automatic robotic testing can reduce the dependence on the internal information of apps. However, capturing GUI element information accurately and effectively from a black-box perspective is a critical issue in robotic testing. This study introduces object detection technology to achieve the visual identification of mobile app GUI elements. First, we consider the requirements of test implementation, the feasibility of visual identification, and the external image features of GUI comprehensively to complete the reasonable classification of GUI elements. Subsequently, we constructed and optimized an object detection dataset for the mobile app GUI. Finally, we implement the identification of GUI elements based on the YOLOv3 model and evaluate the effectiveness of the results. This work can serve as the basis for vision-driven robotic testing for mobile apps and presents a universal approach that is not restricted by platforms to identify mobile app GUI elements.

## 1. Introduction

Mobile app refers to modern user-oriented software that relies on an event-driven graphical user interface (GUI) system (e.g., Android or iOS) to achieve close interaction with users. A series of testing approaches and tools are based on GUI to verify the availability of apps by imitating user interaction to assure the quality of mobile apps [1, 2].

Currently, widely used mobile app testing approaches can be divided into two categories, namely, automated testing and manual testing [2]. Automated testing approaches, such as random testing, script-based testing, and model-based testing [3], capture the internal information (e.g., event flow, source code, and GUI layout) of the app under test (AUT) and take certain strategies for exploring and testing it. However, although these approaches are performed automatically, they have limitations.

Automated testing approaches do not work smoothly for a large number of cross-platform apps, web-based apps, and hybrid apps. With manual testing, such as exploratory testing and crowdsourced testing, testers can easily solve the shortcomings of automated testing with the help of human vision and generalization ability. However, human labor is limited, expensive, inefficient, and prone to errors. Given this situation, robotic testing approaches [4, 5] for mobile apps have been proposed in recent years. This approach attempts to complement the advantages of automated testing and manual testing.

Figure 1 shows the robotic test environment we designed. It consists of two parts, namely, Test Execution Environment and Test Learning Environment. The test execution environment captures the visual information of the AUT through the camera and guides the robotic arm to complete the execution of test action. The test learning environment implements the learning and training of mobile apps through visual information to generate corresponding test strategies. The ultimate goal of this robotic testing is to achieve an automated testing approach that is akin to human testing. It can cognize and learn mobile apps similar to humans under constant interaction while maintaining automatic characteristics.

There are five milestones to be achieved for this automated robotic testing. First, the robot can obtain app interface information completely through a vision that is similar to that of a human (i.e., identify GUI elements and gain GUI structure). Second, the robot can further understand the meaning of the app interface conveyed by the interface information (i.e., analyze app functions and recognize app scenarios). Third, the robot can associate appropriate processing actions based on the meaning of the app interface (i.e., determine test strategy and generate action sequence). Fourth, the robot can judge the interaction results of actions and the app (i.e., receive response results and detect abnormalities interactively). Fifth, the robot can learn to mine and test multiple types of app functions (i.e., improve test coverage and ensure test quality). However, an important prerequisite for the realization of automated robotic testing is whether the robot can visually interact with the app accurately and effectively.

Thus, this study focuses on solving the first and most essential issue of automated robotic testing, which is the visual identification of mobile app GUI elements. We introduce object detection technology [6, 7], which is analyzed and considered suitable for mobile app testing, to achieve the visual identification of GUI elements. The main contributions are presented as follows: (i) the construction of a dataset for identifying mobile app interface elements, including nine main GUI element categories; (ii) optimization of the YOLOv3 model to be more suitable for mobile app GUI element detection; a cross-platform approach for identifying interface elements and promotion of the improvement of robotic testing.

The remainder of this study is organized as follows.  Section 2 introduces the research background and related work.  Section 3 describes the approach of using object detection to identify mobile app GUI elements for robotic testing.  Section 4 discusses the experiment and evaluation results.  Section 5 presents the conclusion and future work.

## 2. Background and Related Work

### 2.1. Mobile App GUI

A GUI is widely used in software development as an essential means of connecting users and software. Unlike desktop software, mobile apps place new requirements on the GUI design because of the limitations of the screen size (palm-use screen replaces larger computer display) and interaction mode (gestures replace mouse and keyboard) of mobile devices. Mobile app GUI needs to be concise enough to achieve good readability and usability. For example, a tree-structured menu is usually designed to expand layer-by-layer in desktop software but is designed as multiple subpages in mobile apps.

The technical implementation of event-driven GUI in mobile apps uses a view-controller combination. The view is used to reflect the elements that a user can see (e.g., a button on an interface) on the interface, and the controller is used to implement interaction with a user (e.g., a click-action applied to a button will trigger something), such as the view object in Android [8] and the UIView and UIControl objects in iOS [9].

All elements of a single GUI are arranged in a tree structure. A node represents an element, and multiple nodes together form a more complex element (or function). In addition, all GUIs of a mobile app can form a directed graph whose nodes represent the GUI state, and edges represent events. Each channel represents a function of the app that is embodied by a GUI.

Therefore, identifying the views of the GUI and recognizing the events bound to them are crucial for mobile app testing.

### 2.2. Automated Robotic Testing for Mobile App

Mobile devices provide rich interaction, such as gestures, voice, and sensors of gravity, acceleration, and light. Effective test coverage of mobile apps cannot be supported by triggering simulated events alone. Some methods that use robotic arms to realize the interaction process are proposed to enhance the realism of mobile app testing [4, 5].

However, the current robot testing for mobile apps only focuses on test execution to solve the complex interaction and anthropomorphic operation problems of mobile apps. For example, robotic arms are used for testing image rectification [10] and the playback of test actions based on coordinate points [11]. Robots are used only as an execution tool in these methods.

For our purposes, we expect the robot to recognize mobile apps and determine what actions to perform. Therefore, we research the visual identification of mobile apps so that the robot can identify the basic structure of mobile app GUIs similar to a human. On this basis, we believe that robotic testing can further reduce reliance on manual labor.

### 2.3. GUI Element Identification for Mobile App Testing

Mobile app testing includes manual testing and automated testing. For manual testing, the identification of GUI elements is conducted by the human visual system. Automated testing can be divided into three groups based on how the GUI information is obtained.

The first group refers to the system level. These approaches record the coordinate position of the low-level input events at a system level, even at the kernel level for testing purposes. They are usually used for the record–replay testing, such as RERAN [12] and Appetizer [13]. This type of approach focuses on obtaining events directly, and they are strongly coupled with hardware or rely on a customized operating system.

The second group refers to the app level. These approaches obtain the GUI dynamic and static information by reading layout files and source code of apps or native tools based on the platform, such as UIAutomatorviewer [14] provided by Android and XCUITest [15] by iOS. These approaches are applied in different testing techniques, including script-based testing, such as Appium [16] and Espprosso [17]; model-based or model learning testing, such as MobiGUITAR [18] and AMOGA [19]; and record–replay testing, such as SARA [20]. They can capture the events and views from the app's perspective and meet the purpose of testing. However, this type of approach relies heavily on app code or specialized tools and is difficult to support for cross-platform or cross-app testing.

The third group refers to the device level. These approaches capture the GUI information visually and use image processing methods (e.g., pixel- or vector-based image recognition) for element matching during testing. They are generally called visual GUI testing (VGT), such as Sikuli [21] and Eyeautomate [22]. This type of approach can be viewed as black-box testing that only identifies and tests apps based on their external behavior. However, they can only judge the preset images and lack generalization. Hence, they serve more as an alternative approach when the internals of the app cannot be accessed.

Although the current identification approaches promote mobile app testing, they are extremely dependent on platforms, systems, or specific tools. Thus, they cannot be used as a universal GUI element identification approach for robotic testing to test various apps.

### 2.4. Vision Technology Used in Mobile App Engineering

Deep learning technology has shown significant progress in the last years, especially in computer vision [23, 24]. Various types of deep learning-based vision technologies, such as image classification, object detection, semantic segmentation, and image caption, have emerged. Each vision technology is dedicated to bringing intelligence to computers through vision. Currently, vision technology is also exploited to help improve the automation of mobile app engineering.

In the development of mobile apps, convolutional neural network (CNN)-based methods are used to convert a GUI design image (a pure pixel UI image generated by UI designers through image editing software, such as Photoshop or Sketch) into a GUI skeleton (which defines the composition of components and layout of GUI) [25]. A prototype is built directly from app screenshots for similar GUI implementation [26], and whether the GUI of a mobile app is implemented according to its intended design is verified [27].

In the testing and security of mobile apps, the image-based detection of privacy acquisition and malicious behavior has been proposed. CNN is used to directly learn the features of sensitive UI widgets or malware for Android apps subject to the rapid progress of mobile app programming and antireverse engineering techniques [28]. In addition, CNN is combined with testing frameworks, such as Appium, to obtain the meaning of specific icons to optimize testing [29].

Vision technology has already been used in mobile app engineering, but they only solve some specific development or testing issues and cannot support the vision-driven robotic testing for mobile apps effectively.

## 3. Approach Description

In view of the above situation, we implement an approach that identifies GUI elements for mobile app testing visually based on object detection technology. The approach involves three main processing phases, namely, GUI element classification, dataset establishment, and object detection model training. The core issue we want to solve in the GUI element classification phase is how to divide the GUI elements properly and effectively for mobile app testing. The core issue in the dataset establishment phase is how to build an effective dataset that can be used to identify GUI elements accurately. The core issue in the model optimization phase is how to train a correct and applicable object detection model considering the features of mobile app testing and the advantages of object detection. Detailed approach descriptions of these processing phases are provided in this section.

### 3.1. GUI Element Classification

Mobile app operating system vendors provide a wealth of GUI controls to meet diverse app design requirements. Even if one control has multiple control versions in different system versions, although some app functions look the same, they are designed differently. This factor also makes the universal identification of app functions difficult for current automated testing. Therefore, we adopt a visual perspective to classify the controls. We are more concerned with identifying the most basic interactive controls.

Figure 2 shows our intention as an example. We expect to visually identify ImageButton, TextView, and ImageView, which provide direct interaction with users in the form of information display or function triggering while ignoring ToolBar, ListView, and LinearLayout, which are composed of ImageButton, TextView, and ImageView. The reason for this is that these indirect combination controls do not have specific visual features. Thus, they are difficult to identify visually. Besides, the features of these combined controls themselves are determined by the basic controls. Hence, ignoring them in the visual identification stage does not lose their information. Therefore, we can still use the idea of software reverse engineering to mine and infer the entire GUI tree from the basic controls gradually.

The specific strategies for GUI element classification are presented as follows.

First, we remove the container-type controls, such as LinearLayout, RelativeLayout, ToolBar, and RadioGroup. These controls are not interactive, and they play more of a supporting role in GUI design. Second, we expect to identify the most basic controls, and we can classify less commonly used complex controls (e.g., AnalogClock, RatingBar) as ImageView or a combination of a set of ImageButton. Third, we merge certain controls with duplicate appearances. For example, although CheckedTextView is different from RadioButton and CheckBox, distinguishing them visually is not easy. The same goes for SeekBar and ProgessBar, MenuItem, and ImageButton. Although we have made trade-offs in the division of control types, ensuring correct and effective visual identification is the priority goal. As for the judgment of similar controls and complex controls, the use of robotic interaction to improve them is appropriate in the follow-up. Finally, Table 1 provides examples of our categories of mobile app GUI elements.

### 3.2. Dataset Establishment

An effectively labeled dataset of mobile app GUI elements is required to achieve accurate visual identification of GUI elements. The large dataset of mobile app UI information, RICO [30], contains 66k + unique UI screens of 6.7k + Android apps in 27 categories. For each UI, it provides a screenshot and a detailed view hierarchy. We implement automatic labeling of elements based on RICO.

A python program was written to help us convert the view hierarchy files of RICO into the labeled XML files (Pascal VOC data format [31]) needed for object detection. The conversion rules are presented as follows: (i) convert according to the determined GUI element classification, (ii) judge the interface composed of nonstandard controls by the parent class information and remove if still cannot be judged, (iii) remove interfaces that are unsuitable for training, for example, if the entire interface is just one picture or a web, (iv) remove the horizontal screen and non1920×1080 resolution interface to unify the sample data, and (v) remove the overlapped and occluded interfaces; that is, some controls in the interface will be covered by other controls, thereby leading to confusion of labeling.

After completing the conversion work, we find that the proportion of controls is extremely imbalanced through statistics. The original data in Table 2 show the distribution of each element category after conversion. TextView and ImageView are the most widely used controls, and they appear in almost all interfaces. However, fewer controls, such as RadioButton, only need to be used in certain functional scenarios, thereby leading to a sample imbalance issue in the dataset.

We adopt three measures to address the sample imbalance. First, we utilize the Android IDE to generate interfaces that only contain those fewer controls additionally. RadioButton shown in Figure 3(a) and Seekbar shown in Figure 3(b) are taken as examples. We generate them in different styles, locations, and background colors randomly to strengthen their data size. Second, by counting the number of various types of controls in each interface, parts of the interfaces with a high proportion of TextView, ImageView, and Button are removed. Third, an instance-switching method [32] for data augmentation that can switch the labeled objects by judging the similarity of the bounding boxes of objects is used to continue to improve our dataset. We use RadioButton, Switch, SeekBar, CheckBox, and EditText to replace TextView, ImageView, and Button on a scale from high to low. We only keep the replaced interface images to further balance the number of controls.  Figure 4 shows an example of this process. The TextViews of the original interface (Figure 4(a)) are replaced by other controls of similar size to conform to a new interface (Figure 4(b)). Table 2 presents the final distribution of elements of the refined dataset.

### 3.3. Object Detection Model

Testing is a dynamic and real-time process. We believe that object detection is suitable for mobile app testing among the current popular computer vision technologies, including classification, segmentation, and semantics.

First, the processing speed of object detection is much better than other technologies. Second, the bounding box of the object detection result is applicable for the representation of element identification. Third, mobile apps should be easy for fingers to interact with, so interface elements should have a relatively large proportion compared with the entire screen. Moreover, the spacing between elements is clear, and the elements are usually arranged in an orderly manner. These characteristics create the advantages of using visual identification.

Current deep learning-based object detection can be divided into two categories: two-stage detection and one-stage detection [6]. For a two-stage detection, in the first stage, a CNN is used to generate a candidate pool of region proposals (the region in pictures that may contain objects). In the second stage, the other CNN makes class predictions for each region's proposal. One-stage detection applies a single CNN to detect the object region directly and predict the class for all positions of a full image simultaneously. In terms of the two object detection technologies, one-stage detection has a faster speed and can meet real-time detection needs, whereas two-stage detection has better detection performance. Given the advantages of real-time detection in the former, we opt for the state-of-the-art YOLO model as our visual identification model for mobile app GUI elements.

Specifically, we chose the YOLOv3 [33] model that evolved from YOLOv1 [34] and YOLOv2 [35]. The YOLOv3 model absorbs the advantages of many other object detection models, such as clustering to obtain anchor boxes to achieve more accurate bounding box prediction and multiscale prediction methods to achieve more accurate detection of different sized objects. In addition, the YOLOv3 uses a flexible network structure, which can be dynamically adjusted on the balance of real-time and accuracy according to actual usage requirements. Moreover, apart from the performance of YOLO in object detection on photos, it also performs well on artworks [33]. Similarly, paintings, cartoons, and vector graphics are heavily used in mobile apps. A more important reason is that we expect to use the object detection model with mature applications as a basis for robotic testing.

Figure 5 shows the network structure of the YOLOv3 model. It practices a Darknet53 network structure without the fully connected (FC) layer for image feature extraction. In Darknet53, the convolutional (CONV) layers use batch normalization (BN) [36] for regularization to accelerate convergence and avoid overfitting and use Leaky ReLU (Leaky) as the activation function. To achieve better training results in deeper networks, the shortcut is introduced by referring to the residual (Res) network [37]. In terms of output, the prediction across scales is applied for reference to feature pyramid networks (FPN) [38] to enhance the detection of different size objects (output in three scales in Figure 5: 20 × 20, 40 × 40, and 80 × 80). Concatenate and upsample are handled to concatenate the low-level features and the high-level features to enhance the precision of object detection.

During the execution of the robotic testing, the YOLOv3 model identifies and outputs the type and position of the controls contained in the captured UI image. The robotic arm executes the test action based on the output of the YOLOv3 model and the test strategy. A human-like vision-driven robotic test is formed under the continuous interaction between the robot and AUT.

### 3.4. Improvement of the YOLO Model

We find some peculiar issues when using the YOLOv3 directly to identify GUI elements. As shown in Figure 6, some controls are identified separately. CheckBox is identified as ImageView and TextView, and a complete ImageView is identified as multiple ImageViews and TextViews. Although some controls do consist of other elements, they are not the result we expected. Such split detection results can confuse the testing. For example, the combination of ImageView and TextView does not convey the functional meaning of a CheckBox.

This result may be caused by the insufficient fusion of target features and context features. Therefore, in response to the issue, we improved YOLOv3 to further promote the detection precision of these controls with multiple elements. The architecture of the improved YOLO model (YOLOv3-IM) is shown in Figure 7. In YOLOv3, the target prediction is made directly when the multiscale features are obtained. Moreover, we add a bottleneck attention module (BAM) [39] to each branch in the neck part of YOLOv3 to extract the key feature of the target better. In addition, the finer-grained features from the lower layers are used as context features to fuse with the attention-optimized target features from the higher layers. The main idea is to strengthen the fusion of target and context features through attention guidance.

The structure of BAM is shown in Figure 8. It calculates channel attention and spatial attention synchronously. Finally, the BAM is obtained by passing through the activation function sigmoid after element-wise summation of the two attention results. In the feature fusion processing (Figure 9), we upsample the target features to match the size of the context features and then concatenate them.

We use features from higher layers with large receptive fields to locate targets through attention mechanisms and then supplement the details of features from lower layers to achieve more accurate detection of the controls with multiple elements.

## 4. Experiment and Evaluation

### 4.1. Training Details

The proposed detection model YOLOv3-IM is trained and tested on an NVIDIA GeForce RTX 2080 GPU. The details are presented as follows:

- Width and height: the default configuration of YOLOv3 is managed to detect objects with the image resolution of 416 × 416 pixels on the COCO dataset. The image resolution of the RICO dataset exploited to obtain the original data is the screen resolution of a general mobile phone (1920 × 1080 pixels). Width and height are reset to an appropriate value of 960 × 960 by considering accuracy and efficiency.
- Data augmentation: we do not carry out a separate data augmentation work on the dataset and only use YOLOv3's own data augmentation. When generating sample images, we randomly rotate them plus or minus 15 degrees (angle = 15). The saturation changes within the range of 1/2 to 2 times (saturation = 2), the exposure amount changes within the range of 1/2 to 2 times (exposure = 2), and the hue changes within the range of 1/2 to 2 times (hue = 0.1).
- We manipulate the k-means algorithm to calculate the anchor prior to fit our classification of mobile app GUI. The GUI elements classified in mobile apps are more of squares or rectangles with a longer width. The anchor values for the three different scales are clustered as (10, 13, 62, 55, 161, 74), (35, 63, 95, 70, 221, 115), and (112, 120, 279,167, 382, 315).

The loss function of YOLOv3 consists of calculating the error of the predicted position (*x*, *y*), the width and height of the bounding box (w, h), classification, and confidence. For the identification of mobile app GUI elements, relative to element classification errors, missing detection of elements is intolerable, thereby leading to incomplete interface information acquisition or even test case execution failure. Therefore, the accurately predicted position (*x*, *y*) and bounding box (w, h) are critical points for our attention, and they are given higher weight.

The specific loss function is defined as follows:

(1) $$\begin{array}{c} L=\lambda_{coord}\sum_{i=0}^{K\times K}\sum_{j=0}^{M}I_{ij}^{obj}\left(2-w_{i}^{*}h_{i}^{*}\right)\left[{\left(t_{w}-t_{w}^{*}\right)}^{2}+{\left(t_{h}-t_{h}^{*}\right)}^{2}\right.\\ +{\left(\sigma \left(t_{x}\right)-\sigma \left(t_{x}^{*}\right)\right)}^{2}+{\left(\sigma \left(t_{y}\right)-\sigma \left(t_{y}^{*}\right)\right)}^{2}\\ +\lambda_{obj}\sum_{i=0}^{K\times K}\sum_{j=0}^{M}I_{ij}^{obj}\left(-1\right)\left[c_{i}^{*}\log\left(c_{i}\right)+\left(1-c_{i}^{*}\right)\log\left(1-c_{i}\right)\right]\\ +\lambda_{noobj}\sum_{i=0}^{K\times K}\sum_{j=0}^{M}I_{ij}^{noobj}\left(-1\right)\left[c_{i}^{*}\log\left(c_{i}\right)+\left(1-c_{i}^{*}\right)\log\left(1-c_{i}\right)\right]\\ +\lambda_{cls}\sum_{i=0}^{K\times K}\sum_{j=0}^{M}I_{ij}^{obj}\left(-1\right)\left[p_{i}^{*}\log\left(p_{i}\right)+\left(1-p_{i}^{*}\right)\log\left(1-p_{i}\right)\right], \end{array}$$

where <*σ*(*t*_*x*_), *σ*(*t*_*y*_), *t*_*w*_, *t*_*h*_, *c*_*i*_, and *p*_*i*_ > represent the center coordinate and width and height of the predicted bounding box, the confidence of detected object, and the probability of classification, respectively. <*σ*(*t*_*x*_^*∗*^), *σ*(*t*_*y*_^*∗*^), *t*_*w*_^*∗*^, *t*_*h*_^*∗*^, *c*_*i*_^*∗*^, and *p*_*i*_^*∗*^ > are the corresponding ground truth. *I^obj^_ij_* denotes if the object appears in *j*th bounding box in grid *i*. The loss of coordinate is calculated by mean square error. (2 − *w*_*j*_^*∗*^*h*_*j*_^*∗*^) is used as a coefficient to suppress calculation differences caused by different object sizes. The loss of object and class are calculated by binary cross entropy. *λ*_*coord*_, *λ*_*obj*_, *λ*_*noobj*_, and *λ*_*cls*_ are the weights of each loss, which are set to 2, 1, 0.2, and 1, respectively, in our training.

After modifying the above configuration, we use the pretrained model weights of YOLOv3 on the ImageNet dataset as the initial weights. We take a batch size of 8 and 50,000 training steps and set weight decay to 0.0001 to start training with a learning rate of 0.001. The entire training process took 51 hours, and the loss value stagnates at 0.09. In addition, we also complete the training of YOLOv3 and Faster R-CNN as a comparison.

### 4.2. Evaluation Metrics

We adopt the evaluation criteria in PASCAL VOC [31] to evaluate the effectiveness of the identification.

The P-R curve shows the performance of calculating the precision and recall under different confidence thresholds. It is an ideal state that precision and recall are high, but usually, they are opposite. In fact, a low confidence threshold will lead to an increase in recall, and a high confidence threshold will lead to an increase in precision:

(2) $$\begin{array}{c} \text{Precision}=\frac{\text{TP}}{\text{TP}+\text{FP}}, \end{array}$$

(3) $$\begin{array}{c} \text{Recall}=\frac{\text{TP}}{\text{TP}+\text{FN}}, \end{array}$$

where TP denotes the number of identified and correctly classified controls, FP denotes the number of identified but incorrectly classified controls, and FN denotes the number of unidentified controls.

The F1 score is the harmonic mean of precision and recall:

(4) $$\begin{array}{c} F1=2\frac{{\text{Precision}}^{*}\text{Recall}}{\text{Precision}+\text{Recall}}. \end{array}$$

Average precision (AP) is obtained by integrating the area under the P-R curve, which is a comprehensive expression of precision and recall. The mean AP (mAP) represents the average value of AP for each category:

(5) $$\begin{array}{c} \text{Average Precision}=\int_{0}^{1}p\left(r\right)dr, \end{array}$$

(6) $$\begin{array}{c} \text{mAP}=\frac{1}{n}\sum_{1}^{n}\text{AP}. \end{array}$$

Frames per second (FPS) is used to evaluate the detection efficiency, that is, the number of images that can be detected per second.

### 4.3. Dataset Evaluation

In this section, the validity of the established detection dataset for mobile app GUI elements is evaluated. We use the classical one-stage model YOLOv3 and the two-stage model Faster R-CNN to conduct a comparative evaluation on the original dataset and the refined dataset, respectively.

For the experiment's result, the P-R curve of each category detected by YOLOv3 on the original dataset and the refined dataset is shown in Figures 10(a) and 10(c). The P-R curves of the two models on the original dataset and the refined dataset are shown in Figures 10(b) and 10(d). The comparative results of the two models are exhibited in Table 3.

As seen from the results, the refined dataset improves the mAP of YOLOv3 and Faster R-CNN by 17.95% and 13.17%, respectively. In addition, the average precision of the categories with small data amounts, such as RadioButton, CheckBox, and EditText, has significantly improved.

Although the mAP of Faster R-CNN is slightly higher than YOLOv3, the FPS of Faster R-CNN is much lower than that of YOLOv3. Therefore, YOLOv3 can support a broader range of test requirements, such as the fast test execution and the capture of the real test process, whereas Faster R-CNN can be more of an alternative.

### 4.4. Approach Evaluation

In this section, we compare the GUI identification effect of the improved YOLOv3-IM with other models.  Table 4 shows the comparison results. Compared with YOLOv3, YOLOv3-IM has improved in precision, recall, mAP, and F1. The mAP of YOLOv3-IM finally reaches 85.50%, which is 5.3% higher than YOLOv3.

Figure 11 shows the comparison detection examples of YOLOv3 and YOLOv3-IM. The improvement of YOLOv3-IM is mainly reflected in (i) the correct identification of composite controls, such as CheckBox, RadioButton, and EditText, (ii) complete identification of multielement controls, such as large text and element-rich images, (iii) the positioning of the bounding box is more accurate, and (iv) the missed detection of some small elements has also been improved under the attention mechanism.

The object detection model is flexible in use. According to different usage scenarios, parameters, such as confidence and IOU, can be adjusted to achieve suitable detection. For example, in some test situations that do not require precise classification, the confidence can be ignored to achieve high-performance single-object detection.

Although we have improved the precision of detection of mobile app GUI elements, some points are still worth discussing. To provide the identification effect of each category more clearly, we calculate and express the detected results of the YOLOv3-IM model in the form of a confusion matrix in Table 5.

For the text controls, some ImageViews and Buttons are still incorrectly recognized as TextView. Some button controls with inconspicuous borders and some text with artistic fonts confuse the identification of TextView. In particular, no obvious difference is observed between TextView and clickable text buttons in some apps. They are difficult to distinguish by image features alone. Perhaps the addition of text semantic recognition will improve it.

For image controls, the identification difficulty lies in the feature differences between images. Compared with SeekBar and Switch, which have more fixed styles, ImageView has more mutual error detection because of their rich styles. Moreover, some suggestive icons are very similar to ImageButtons.

Furthermore, some controls leave more blank parts because we label the bounding box of elements completely based on the size of the control but not the content of the control. This may cause the short text to be not well included.

The experiment results demonstrate that the mobile app GUI elements can be properly identified in most cases. Regarding the shortcomings, at the object detection level, subsequent further optimization of the object detection model, the expansion of data samples, and the subdivision of GUI element categories are effective ways to strengthen the identification effect. However, we have obtained a relatively high object detection precision [7]. Further optimization of object detection results may be complicated and of high cost.

In addition, relying solely on visual technology cannot fully realize the identification and understanding of mobile app GUI elements. Judging the meaning and purpose of some controls and even some interfaces based on visuals alone is difficult. For automated robotic testing, the object detection technology will be used more as a trigger to begin the robot's exploration of apps. Combined with testing, continually interacting with apps to obtain feedback information and even construct domain models based on visual information with functional scenarios as the objects may further promote the revision of the identification results and the understanding of mobile app GUI's representative meaning at the test level.

### 4.5. Threats to Validity

We conclude the potential threats to the validity in the experiment as the following aspects:

- Uncertainty in the classification of GUI elements: different from the detection of natural objects (e.g., a tree or a cat), differences may exist in the visual identification of GUI elements from software and user perspectives. For an interface, software engineers can observe the composition of controls, but ordinary users may see the composition of text and images. Therefore, classifying the controls visually better needs to be decided according to the purpose of use. In our experiment, we selected and merged the control categories. We cannot say that it is completely appropriate, but we attempt to achieve a balance between the difficulty of implementation and the effect of identification. We will further clarify the meaning of interface elements, interface areas, and even the entire interface through element combinations and interactive judgments.
- Rich diversity of GUI elements: current mobile apps are still in rapid development. The styles and categories of controls and even how they are used are likely to continue to be added or improved. The game app also has a unique control style. The diversity of mobile apps makes the covering of all GUI features difficult, although RICO has collected a considerable number of apps in different categories. Thus, we believe that ensuring the validity of identification is a continuous task. However, a transfer learning strategy can be adapted to expand the adaptability to the diversity of elements. The model can be fine-tuned on a small new sample dataset (GUI samples containing new control categories or styles) to quickly achieve effective results based on our existing object detection neural network weights.
- Merging some GUI element categories: in the establishment of our dataset, the merging of control types is a compromise strategy that we have adopted. Given the difficulty of the visual identification of some elements, their features are too variable, or the sample size is very sparse. In addition, compared with obtaining accurate app definitions from the code, the app information provided by an interface image has limitations and uncertainties. Moreover, the definition of controls is very flexible. Whether some controls are bound to actions, such as long press, double click, or swipe, is even difficult to judge only visually. Therefore, repeated interaction is still essential to realize the cognition of the app from a black-box perspective.

## 5. Conclusion

In this study, we adopt object detection technology to identify mobile app GUI elements to support the realization of automated robotic testing (a testing approach that combines the advantages of manual testing and automated testing). The final identification result reaches a relatively high precision. It provides a means of universal identification for robotic testing. For future works, we will use the interactive judgment between the robot and mobile apps to further improve and revise the identification results while enhancing the identification accuracy through sample expansion and algorithm optimization. Meanwhile, an online website for the entire robotic testing project is already under consideration. For GUI element identification, it will provide online viewing, downloading, and supplementation of datasets, as well as online GUI interface identification and result file generation. Furthermore, the aforementioned work will be the basis for robotic testing to cognize the meaning of mobile app GUI.

## Figures and Tables

**Figure 1:** Robotic test environment for mobile app testing.

**Figure 2:** GUI controls expected to be identified.

**Figure 3:** Generated interfaces to enhance data size. (a) Generated interface of RadioButton. (b)Generated interface of SeekBar.

**Figure 4:** Balance the dataset by instance-switching. (a) Original interface. (b) Processed interface.

**Figure 5:** YOLOv3 used for robotic test execution.

**Figure 6:** Split detection results by YOLOv3 (CheckBox is detected as ImageView and TextView; ImageView is detected as ImageView and TextView).

**Figure 7:** Architecture of the proposed YOLOv3-IM for GUI element detection.

**Figure 8:** Bottleneck attention module (BAM) architecture.

**Figure 9:** Feature fusion processing.

**Figure 10:** P-R curves of the detection of mobile app GUI elements. (a) P-R curves of each category detected by YOLOv3 on the original dataset. (b) P-R curves of the two models on the original dataset. (c) P-R curves of each category detected by YOLOv3 on the refined dataset. (d) P-R curves of the two models on the refined dataset.

**Figure 11:** Identification results of mobile app GUI elements.

**Table 1:** Categories of GUI elements.

Categories	GUI elements
TextView	
EditText	
Button	
Switch	
RadioButton	
CheckBox	
ImageView	
ImageButton	
SeekBar	

**Table 2:** Distribution of elements in the dataset.

Categories	Original data	Generated data	Data balance	Total
TextView	233,411	0	−216,181	17,230
ImageView	107,230	0	−90,441	16,789
Button	50,680	0	−34,690	15,990
ImageButton	8,798	2,500	3,844	15,142
EditText	7,356	3,500	41,47	15,003
CheckBox	5,936	4,500	5,237	15,673
SeekBar	1,971	6,000	6,253	14,224
Switch	1,784	6,000	7,013	14,797
RadioButton	408	6,000	7,604	14,012

**Table 3:** Results of the detection on the datasets (IOU > 0.5).

Dataset	Model	Average precision (%)									mAP (%)	FPS
		Button	CheckBox	EditText	ImageButton	ImageView	RadioButton	SeekBar	Switch	TextView		
Original dataset	YOLOv3	65.74	39.23	46.74	70.95	61.03	42.45	80.31	85.25	68.54	62.25	26
	Faster R-CNN	67.90	48.63	56.44	75.38	65.76	57.57	82.23	86.95	72.63	68.16	0.25
Refined dataset	YOLOv3	74.09	86.71	86.62	79.54	64.26	86.43	83.29	87.87	72.95	80.20	26
	Faster R-CNN	74.58	87.96	86.67	81.03	76.65	86.49	84.12	89.66	73.70	81.33	0.25

**Table 4:** Comparison of results from different models (IOU > 0.5) (%).

Model	Precision	Recall	mAP	F1	FPS
Faster R-CNN	80.67	81.36	81.33	80.42	0.25
YOLOv3	79.28	82.85	80.20	79.59	26
YOLOv3-IM	86.63	84.97	85.50	84.53	22

**Table 5:** Confusion matrix for detected results (confidence >0.8, IOU > 0.5) (%).

Categories	TextView	ImageView	Button	ImageButton	EditText	CheckBox	SeekBar	Switch	RadioButton
TextView	81.8	0.9	8.6	0	4.4	7.1	0	0	4.7
ImageView	1.1	78.5	0.6	5.1	0	0	8.1	6.2	0
Button	8.2	1.2	83.6	0.3	0.6	4.1	0	0	3
ImageButton	0.5	8.7	3.4	84.6	0	0	2.1	4.5	0
EditText	0.1	1.2	0.9	0.1	87.2	0.8	0	0	0
CheckBox	0.8	2.3	0.3	0	0.8	88.2	0	0	0
SeekBar	0	4.6	0	1.3	0	0	87.9	0.1	0
Switch	0	1.4	0	2.8	0	0	1.5	88.9	0
RadioButton	0.6	0.3	0.3	0	0.9	0	0	0	88.5

*Note*. The caption of the first row represents the identified control categories, and the first column represents the actual control categories.

## Data Availability

The data used to support the findings of this study are available from the corresponding author.
